# Berberine Attenuates IL-1*β*-Induced Damage of Nucleus Pulposus Cells *via* Activating the AMPK/mTOR/Ulk1 Pathway

**DOI:** 10.1155/2022/6133629

**Published:** 2022-07-23

**Authors:** Liaoyuan Huang, Jianming Chen, Danhai Wu, Kan Wang, Weigang Lou, Jianmin Wu

**Affiliations:** ^1^Department of Orthopedics, Ningbo No.6 Hospital, Ningbo City, Zhejiang Province 315040, China; ^2^Department of Radiology Emergency, Ningbo No.6 Hospital, Ningbo City, Zhejiang Province 315040, China; ^3^Department of Radiology, Ningbo No.6 Hospital, Ningbo City, Zhejiang Province 315040, China

## Abstract

Intervertebral disc degeneration (IDD) is a chronic progressive condition mainly caused by excessive inflammatory cytokines. Berberine (BBR) exerts anti-inflammatory effect on diseases and protective effect against IDD. However, the mechanism is not uncertain. This study is aimed at investigating the molecular mechanism of BBR on IDD. Nucleus pulposus (NP) cells were treated with BBR at different concentrations. The IDD rat model was established by acupuncture. The effect of BBR on interleukin- (IL-) 1*β*-induced cell proliferation was measured by CCK-8 assay and BrdU staining. The role of BBR in IL-1*β*-induced apoptosis, autophagy repression, and extracellular matrix (ECM) degradation was measured by Annexin/PI staining, immunofluorescence, and immunoblot. The effect of BBR on IDD was investigated in rat. Our findings showed that BBR restored cell growth and attenuated apoptosis in IL-1*β*-induced NP cells. BBR also prevented the IL-1*β*-induced ECM degradation through regulating ECM-related enzymes and factors. Additionally, BBR significantly activated autophagy repressed by IL-1*β*. Autophagy stimulated by BBR was diminished by the inhibition of the AMPK/mTOR/Ulk1 signaling pathway. *In vivo* study also showed BBR attenuated intervertebral disc degeneration. BBR could attenuate NP cells apoptosis and ECM degradation induced by IL-1*β* through autophagy by the AMPK/mTOR/Ulk1 pathway. This study suggests BBR might function as an AMPK activator to alleviate IDD progression.

## 1. Introduction

Intervertebral disc degeneration (IDD) is a common clinical condition and usually resulting in neck or back pain [1]. The process of IDD is often considered abnormal and cell-mediated responses to progressive structural failure as a result of aging, genetic alterations, and some environmental factors [1, 2]. The intervertebral disc mainly contains annulus fibrosus (AF), nucleus pulposus (NP), and cartilage endplates. Extracellular matrix (ECM), produced by NP cells, is the main component of gelatinous tissue in NP. Various pathological processes are involved in IDD, including ECM degradation and excessive apoptosis of NP cell [3]. Inflammation process is commonly regarded as critical events during IDD, mediated by inflammatory cytokines, such as tumor necrosis factor- (TNF-) *α* and interleukin- (IL-) 1*β* [4]. IL-1*β* has been proven to be the main cytokine overexpressed in IDD tissues and associated with pathological activities of NP cells, such as matrix catabolism, oxidative stress, inflammatory response, and cell apoptosis [4, 5]. Thus, mediation of IL-1*β* expression in NP cells might be a potential approach to prevent or alleviate IDD.

There are three major forms of cellular death: apoptosis, autophagy, and necrosis [6]. Autophagy is identified as a stress-mediated process engulfing dysfunctional proteins, organelles, and pathogens into autophagosome [7]. As reported, autophagy can enhance cell survival and serve as an essential role in development of different diseases [8], such as Alzheimer's disease [9], osteoarthritis [10], and cancer [11]. Previous studies have demonstrated that autophagy could protect NP cells from excessive apoptosis [12–14]. Adenovirus-Mfn2 injection ameliorated the development of IVDD in rats; besides, further mechanism investigation showed that the inhibition of autophagy suppressed the protective effect of Mfn2 overexpression on NP cells, aggravating mitochondrial dysfunction and cellular apoptosis [15]. Quercetin enhanced the expression of SIRT1 and autophagy; however, autophagy inhibitor 3-MA reversed the protective effect of quercetin on apoptosis and ECM degeneration in NP cells, suggesting induced autophagy alleviated the progression of IDD [16]. Most studies indicate that activated autophagy slows down the progression of IDD [17]. Hence, we hypothesized that autophagy might be involved in the development of IDD.

Berberine (BBR, C_20_H_18_NO_4_) is an ammonium salt belonging to a group of benzylisoquinoline alkaloids isolated from *Berberis* species. Berberine shows a molar weight of 336.36 g/moL and a melting point of 145°C [18]. BBR exhibits diverse medical potentials, including anti-inflammation and antivirus [19]. Emerging study reveals that BBR can induce autophagy in a variety of cells [20]. Besides, more recent studies suggest that BBR might impede the progression and development of osteoporosis [21], osteoarthritis [22], and rheumatoid arthritis [23] *via* different signaling pathways, such as p38/MAPK, AMPK, Wnt/*β*-catenin, PI3K/Akt, NF-*κ*B as well as oxidative stress signaling [24, 25]. Moreover, BBR is reported to suppress cell apoptosis, ECM degradation, and oxidative stress by activating autophagy in NP cells [26]. However, the underlying mechanism has not been well investigated. Hence, the current research is aimed at studying the effect and molecular mechanism of BBR in cell viability, apoptosis, ECM degradation, and autophagy in IL-1*β*-induced rat NP cells and a rat IDD model.

## 2. Material and Methods

### 2.1. Reagent

Berberine is an isoquinoline quaternary alkaloid isolated from numerous medicinal herbs of the genera *Berberis*. Berberine (purity > 98.5%), 3-MA (3-methyladenine, autophagy inhibitor), and IL-1*β* were purchased from Sigma (USA). And dorsomorphin (compound c, CC, AMPK inhibitor) was obtained from APExBIO Technology (USA).

### 2.2. NP Cells Culture

NP cells were first isolated from SD rats described elsewhere [27]. In short, SD rats (330-370 g) were euthanized with an overdose of 800 mg/kg sodium pentobarbital. Under aseptic conditions, the spinal columns from L1 to L5 were carefully removed. Gel-like nucleus pulposus tissues were then separated and washed with sterile normal saline solution and digested by 0.1% collagenase and 2 U/mL hyaluronidase for 4 h at 37°C. Then the samples were transferred to DMEM (Invitrogen, USA) with 10% fetal bovine serum (FBS; Invitrogen, USA) supplemented with 1% penicillin-streptomycin solution (Sigma-Aldrich, St. Louis, MO, USA) and incubated at 37°C with 5% CO_2_. NP cells grew out from the tissues after about 1 week. When confluence reached 85%, the cells were subcultured and used for subsequent experiments.

### 2.3. CCK-8 Assay

CCK-8 assay was used to detect the cell viability of NP cells. Briefly, NP cells were seeded in 96-well plates with a density of 2.5 × 10^5^ and incubated for 24 hours at 37°C with 5% CO_2_. Subsequently, CCK-8 reagent (10 *μ*L) was added to each well, and the cells were cultured at 37°C for another 1 h. The optical density of solution was detected at 490 nm using a microplate reader (Thermo Electron Corp, Waltham, MA, USA).

### 2.4. BrdU Assay

BrdU assay (Roche, USA) was conducted to determine the cell proliferation. At first, NP cells were cultured in DMEM with 10 *μ*M BrdU for 1 h. Then cells were fixed in 4% paraformaldehyde for 15 min, washed with phosphate-buffered saline (PBS) buffer, and incubated with a primary antibody against BrdU for 1 h at 37°C, followed by PBS buffer washing for three times. Subsequently, the cells were incubated with secondary antibody for another 1 h at room temperature. BrdU-positive cells were calculated by a microscopy.

### 2.5. Flow Cytometry Analysis of Cell Apoptosis

Treated NP cells were suspended in PBS at 4°C, followed with centrifugation for 5 min. The supernatant was discarded, and NP cells were collected. Subsequently, the NP cells were gently resuspended in 300 *μ*L of binding buffer and adjusted to a final concentration of 1 × 10^6^/mL. Next, cell suspension of 100 *μ*L was added to the tube, supplemented with 5 *μ*L of FITC-labeled Annexin V and 10 *μ*L of PI solution. The samples were incubated in dark for 20 min and added with 400 *μ*L of binding buffer. Finally, the ratio of apoptotic cells was detected by a CytoFLEX LX Flow Cytometer (Product No.: A21000090, Beckman Coulter), and the results were analyzed with the FlowJo software (BD, USA).

### 2.6. Immunofluorescence

Immunofluorescence assay was performed to analyze the expression of collagen II and LC3. NP cells were fixed in 4% paraformaldehyde, washed by PBS buffer with Triton X-100 for 10 min, and blocked in PBS buffer containing 5% bovine serum (BSA) for 20 min. Subsequently, the samples were incubated with primary antibodies overnight at 4°C, followed with incubation of fluorescein isothiocyanate- or tetramethyl rhodamine isothiocyanate-conjugated second antibodies for 1 h. The slices were then labeled with DAPI (Thermo Fisher, USA) for 5 min and observed under a microscope. Primary antibodies against LC3 and collagen II were purchased from Invitrogen (USA).

### 2.7. Immunoblot

NP cells or rat tissues were lysed using radioimmunoprecipitation assay RIPA buffer (Beyotime, China), and the protein amount was quantified using protein assay reagent (Bio-Rad, Mississauga, Canada). A total of 20 *μ*g protein of each sample was loaded with 10% sodium dodecyl sulfate-polyacrylamide gel electrophoresis (SDS-PAGE) and transferred to the PVDF membrane (Bio-Rad, USA), blocking with 5% nonfat milk in TBST buffer. Then the membranes were incubated with primary antibodies at 4°C overnight, followed with incubation of corresponding secondary antibodies for 1 h at room temperature. Primary antibodies used were as follows: anti-collagen II antibody (ab188570, 1/1000), anti-Cleaved Caspase-3 antibody (ab32042, 1/500), anti-Cleaved-PARP1 antibody (ab32064, 1/1000), anti-PCNA antibody (ab18197, 1 *μ*g/mL), anti-MMP13 antibody (ab39012, 1/3000), anti-Beclin 1 antibody (ab210498, 1/1000), anti-LC3A/B antibody (ab62721, 1 *μ*g/mL), anti-p62 antibody (ab240635, 1/1000), anti-AMPK*α* (ab187408, 1 *μ*g/mL), anti-p-AMPK*α* (ab133448, 1/1000), anti-mTOR antibody (ab134903, 1/10000), anti-mTOR (phospho S2481) antibody (ab137133, 1/1000), anti-ULK1 antibody (ab240916, 1/1000), anti-ULK1 (phospho S556) antibody (ab203207, 1/100), and anti-GAPDH antibody (ab8245, 1/500) were all purchased from Abcam (Cambridge, MA, USA), and anti-aggrecan antibody (#MBS9383447, 1.0 mg/mL) were purchased from BioSource (Camarillo, CA, USA). The bands were detected with electrochemiluminescence reagent (Beyotime, China), and the intensities were analyzed with the ImageJ software.

### 2.8. RNA Extraction and Reverse Transcription-Quantitative PCR (RT-qPCR)

Total RNA was extracted from treated NP cells as described using RNAiso Plus (Takara, Japan), and cDNA was synthesized using the Prime Script RT Master Mix kit (Takara, Japan) according to the manufacturer's manual. The mRNA expression was detected using SYBR green Mix (Takara, Japan) in an Exicycler™ 96 (Bioneer Corporation, Daejeon, Korea). PCR reaction conditions were as follows: initial activation step at 95°C for 15 min, followed by 40 cycles, denaturation at 94°C for 15 s, annealing at 55°C for 30 s, and extension at 72°C for 30 s. GAPDH was used as an internal control. Relative RNA levels were calculated by the 2^-*ΔΔ*Ct^ method. The primers used were listed as follows [28]: aggrecan (F 5′-GTCAGGTACCCCATCCACAC-3′ and R 5′-TCTGCGAAGCAGTACACGTC-3′); MMP-13 (F 5′-GTGACAGGAGCTAAGGCAGA-3′ and R 5′-AGCATGAAAGGGTGGTCTCA-3′); type II collagen (F 5′-CAAGAAGGCCTTGCTCATCC-3′ and R 5′-CAGTGTACGTGAACCTGCTG-3′); and GAPDH (F 5′-CGCGGTTCTATTTTGTTGGT-3′ and R 5′-CTTCAAACCTCCGACTTTCG-3′).

### 2.9. IDD Rat Model

IDD rat models were established by annulus fibrosus (AF) puncture surgery as described elsewhere [12, 23]. In brief, the rats were anaesthetized by 30 mg/kg body weight pentobarbital sodium through intraperitoneal injection (i.p.). The needle of 4 mm in length (27 G) was used to puncture the whole layer of AF though the tail skin perpendicularly. Before extraction, the needle was rotated 360° and stayed in position for 1 min. The sham group only received skin incision and suture.

### 2.10. Animal Treatments

A total number of 30 Sprague Dawley rats (200~250 g, male, aged 2 months, 10 per group) were randomly grouped: (1) sham group was i.p. injected with normal saline; (2) IDD group; and (3) IDD + BBR group. The IDD group and IDD + BBR group underwent AF puncture surgery. BBR (in normal saline, 150 mg/kg) was administered intragastrically in the BBR group. An equal amount of normal saline solution was intragastrically given to the IDD group. All the treatment started after operation and last until sacrifice.

All the *in vivo* experiments had obtained approval from the Ethics Review Committee of Ningbo No.6 Hospital.

### 2.11. Immunohistochemical Examination

Rat tissues were fixed with formaldehyde, embedded by paraffin, and then sectioned. The samples were stained with Hematoxylin Eosin (H&E) followed with safranin O-fast green(S-O) (Sigma, USA). The cellularity and morphology of NP and AF were detected using a microscope and evaluated by a grading scale [29].

### 2.12. Terminal Deoxynucleotidyl Transferase (TdT) dUTP Nick-End Labeling (TUNEL) Assay

The slides were used for TUNEL assay (Abcam, USA) to evaluate cell apoptosis in rat tissues under a microscope.

### 2.13. Statistical Analysis

Statistical analyses were performed using the GraphPad Prism 8 software. Quantitative data are presented as mean ± standard deviation (SD). Comparison between two groups was performed using the Student *t*-test. Comparison among three or more groups was conducted using the one-way analysis of variance (ANOVA) followed by Tukey's post hoc test. Differences were considered significant if *P* < 0.05.

## 3. Results

### 3.1. Berberine Promotes Cell Proliferation and Suppresses Apoptosis in IL-1*β*-Induced NP Cells

To evaluate the cytotoxicity of BBR on NP cells, the viability of NP cells was measured. As shown in Figure 1(a), cell viability was significantly decreased upon BBR treatment above 2 *μ*M on 7 days posttreatment, suggesting BBR has no cytotoxicity to NP cells at a concentrations less than 2 *μ*M. Subsequently, the optimal concentration of BBR for IL-1*β*-induced NP cells was measured. As shown in Figure 1(b), IL-1*β* treatment obviously decreased cell viability, which was restored by BBR at a concentrations above 0.5 *μ*M on 4 days and 6 days posttreatment. Therefore, a concentration of 1 *μ*M for BBR was selected for the following investigations.

Next, the effect of BRR on cell proliferation and apoptosis in IL-1*β*-induced NP cells was investigated. The cell growth was markedly repressed by IL-1*β*, and BBR treatment attenuated the inhibitory effect of IL-1*β* on cell growth (Figure 1(c)). The number of BrdU-positive cells in control was around 4-fold over that in IL-1*β*-induced cells, while BBR treatment increased the number of BrdU-positive cells by 3-fold compared to IL-1*β*-induced cells (Figures 1(d) and 1(e)). Since NP cell apoptosis plays a critical role in IDD progression, the effect of BBR on cell apoptosis was examined. It showed IL-1*β* increased apoptotic ratio to up to around 3.8-fold compared to the control, which could be recused by cotreatment with BBR (Figures 1(f) and 1(g)). Besides, Cleaved Caspase-3 and Cleaved-PARP were upregulated, and PCNA was downregulated in IL-1*β*-induced NP cells; nevertheless, the effect of IL-1*β* was reversed by BBR treatment (Figures 1(h) and 1(i)). All these results indicated that Berberine promoted cell proliferation and suppressed apoptosis in IL-1*β*-induced NP cells.

### 3.2. Berberine Suppresses ECM Degradation in IL-1*β*-Induced NP Cells

To investigate the effect of BBR on ECM degradation in IL-1*β*-induced NP cells, the expressions of ECM-related factors were detected. The findings revealed IL-1*β* treatment remarkably reduced mRNA levels of collagen II and aggrecan in IL-1*β*-induced cells by 5- and 2-fold than controls, respectively, which were recovered by BBR treatment. Moreover, MMP-13 mRNA expression in IL-1*β*-induced NP cells was about 6-fold over the control but attenuated by BBR treatment (Figure 2(a)). The results of western blot for protein were consistent with the detection of qRT-PCR (Figure 2(c)). Immunocytochemistry also showed that IL-1*β* markedly inhibited the synthesis of collagen II, whereas this effect was reversed by BBR treatment (Figure 2(b)). These findings suggested that BBR suppressed ECM degradation in IL-1*β*-induced NP cells.

### 3.3. Berberine Activates Autophagy in NP Cells

BBR was reported to enhance autophagy in various cells [16]. The regulation of BBR for autophagy in IL-1*β*-induced NP cells was detected. As shown in Figures 3(a) and 3(b), compared to the controls, Beclin1 expression and LC3II/LC3I ratio in IL-1*β*-treated cells were reduced 5- and 4-fold, respectively, and p62 expression was increased around 9-fold. The effect of IL-1*β* on autophagy in NP cells was partly reversed by BBR (Figures 3(a) and 3(b)). We also observed that 3-MA rescued the effect of BBR on the expression of proteins related to autophagy in cells treated by IL-1*β*. In addition, the immunocytochemistry of LC3 staining suggested that autophagosomes was increased by BBR in NP, conversely blocked by 3-MA treatment (Figure 3(c)). All these results illustrated that BBR activated autophagy in NP cells.

### 3.4. Berberine Regulates Autophagy and Cell Apoptosis by Activating the AMPK/mTOR/Ulk1 Signaling Pathway in NP Cells

Previous studies demonstrated that BBR induced autophagy through various signaling pathways, including AMPK and mTOR [24]. In glioblastoma cells, BBR was reported to induce autophagy *via* targeting the AMPK/mTOR/ULK1 pathway [30]. Thus, we hypothesized that BBR might activate autophagy through the AMPK/mTOR/ULK1 signaling pathway in IL-1*β*-induced NP cells. As shown in Figures 4(a) and 4(b), BBR significantly enhanced the phosphorylation of AMPK*α* and LC3II/LC3I ratio and increased the protein levels of Beclin1 and PCNA but reduced phosphorylation levels of mTOR and Ulk1 as well as elevated protein levels of p62, Cleaved Caspase-3, and Cleaved-PARP. However, CC treatment obviously inhibited the regulation of BBR for the MPK/mTOR/ULK1 pathway and protein expression related to autophagy and cell apoptosis. All the results revealed that BBR regulated autophagy and cell apoptosis by activating the AMPK/mTOR/Ulk1 signaling pathway in NP cells.

### 3.5. Berberine Ameliorates Intervertebral Disc Degeneration *In Vivo*

To evaluate the effect of BBR on intervertebral disc degeneration *in vivo*, an IDD rat model was used (described above). A total of 30 SD rats were divided into three groups (200-250 g, male, aged 2 months, *n* = 10 for per group). The staining of disc samples showed that the discs are mainly stellar-shaped and evenly surrounded by abundant ECM in the sham group (Figure 5(a)). In the IDD group, NP cells in tissues tended to cluster and separated by wispy proteoglycan matrix. However, the degeneration of proteoglycan matrix was attenuated by BBR treatment, and the morphology of NP cells was maintained (Figure 5(a)). In addition, the histological score of the BBR + IDD group was markedly lower than that of the IDD group (Figure 5(b)). BBR suppressed cell apoptosis by 2-fold in the IDD group (Figure 5(c)). Besides, AMPK*α* phosphorylation, conversion of LC3 I to LC3 II, and collagen II expression were alleviated in IDD rats; meanwhile, Cleaved-PARP expression was elevated. Compared to the IDD group, BBR was found to aggravated AMPK*α* phosphorylation, conversion of LC3 I to LC3 II, and upregulated collagen II expression but suppressed Cleaved-PARP (Figures 5(d) and 5(e)). The above findings illustrated that BBR attenuated intervertebral disc degeneration in IDD rats.

## 4. Discussion

IDD is a chronic and progressive disease mainly caused by neck or back pain [3]. In the last decades, the treatment of IDD is costly but relatively ineffective [2]. Therefore, it is of great significance to comprehensively find out the cellular biology and underlying molecular mechanism of IDD. Intervertebral disc is a unit compromised of peripheral AF, central NP, and cartilage end plates, contributing to the flexibility, motion, and weight bearing of spine. Chondrocyte-like rounded cells are the main NP cells in adults, ECM in NP mainly consists of type II collagen and proteoglycan, and aggrecan belongs to one of the most common proteoglycan [31]. As we know, the decrease of viable cells and alteration of cell phenotype are the most important parts during the pathological process of IDD [32], such as cell death, proliferation, and senescence [2]. The changes in cell viability and phenotype led to alterations in the production of ECM, inflammatory cytokines, and degradative enzymes [3, 33]. Inflammatory cytokines, such as TNF-*α* and IL-1*β*, exacerbated inflammatory process and ECM degradation and activated various singling pathways during IDD [4]. As reported, IL-1*β* overexpression was closely associated with the development of IDD [34] and enhanced the expression of matrix metalloproteinases, leading to ECM degradation [35]. Besides, IL-1*β* induced NP cells apoptosis and promoted IDD progression [36]. In this study, we employed IL-1*β* to stimulate rat NP cells to establish a model of IDD *in vitro*.

BBR is a natural compound mainly extracted from Berberidaceae family. Several studies have illustrated the multiple biological activities of BBR, including antihypertense, anti-inflammation, and anticancer [18]. As reported, BBR accelerated cell death in KB oral cancer *via* apoptotic signaling pathways [37]. BBR is also found to promote the apoptosis of liver cancer cells through the mitochondrial pathway [38], whereas BBR exhibits antiapoptotic effects on some other diseases. A recent study reported that BBR plays a protective role in acute liver failure *via* inhibiting inflammatory cytokine production and mitochondria-dependent apoptosis [39]. Additionally, BBR suppressed apoptosis and ECM degradation in NP cells [12]. In this study, we also found BBR suppressed apoptosis and ECM degradation in NP cells. Type II collagen and aggrecan are considered the main component of ECM in NP [31]; meanwhile, MMP-13 is the main protease degrading type II collagen and aggrecan [40]. Our results revealed that BBR treatment increased the expression of collagen II and aggrecan but decreased MMP-13 expression in NP cells. We further found that BBR enhanced cell viability and suppressed cell apoptosis as well as ECM degradation in IL-1*β*-induced NP cells. These results are consistent with most previous studies.

Autophagy is a critical process providing needed metabolites to cells by degrading unnecessary proteins and organelles and plays a role of double-edged sword in diseases development by either promoting cell survival or causing cell death [6]. It contributed to accelerating cell death and enhancing cell survival under stresses, such as cell starvation and endoplasmic reticulum stress [7]. Autophagy also plays critical roles in musculoskeletal disorders, including IDD and osteoarthritis [10, 41]. Based on the analysis of the difference between healthier discs and degenerated discs, it was found that autophagy-related genes were highly expressed in degenerated discs [41]. Moreover, a previous study illustrated that activation of autophagy inhibited apoptosis of chondrocytes and NP cells induced by inflammatory reaction *via* suppressing NF-*κ*B and JNK signaling pathways [42]. BBR, an autophagy modulator, has been reported to induce autophagy in different systems through various signaling pathways, including mTOR, JNK, and p38/MAPK [20]. However, up to now, limited researches focus on the role of BBR in autophagy. A previous study reported that BBR induced autophagy in NP cells through inhibiting the NF-*κ*B pathway [28]. In the present study, we for the first time demonstrated that BBR treatment might activate autophagy in IL-1*β*-induced rat NP cells. Besides, BBR serves as an AMPK activator in different diseases. In glioblastoma cells, BBR promoted autophagy through activating the AMPK/mTOR/Ulk1 signaling pathway [30]. BBR induced AMPK-dependent activation of Nrf2 in LPS-stimulated macrophages and endotoxin-shocked mice [43]. A review also demonstrates that AMPK and its activator BBR can suppress oxidative stress, neuroinflammation, mitochondrial disorder, apoptosis, and autophagy disorder in neurodegenerative disorder [44]. Emerging evidence showed miR-143-5p targeted eEF2 to promote IDD progression through activating the AMPK signaling pathway in NP cells [45]. All these researches indicate that BBR might activate the AMPK signaling pathway in IDD. Consistent with previous studies, our study found that BBR regulated autophagy and cell apoptosis through activating the AMPK/mTOR/Ulk1 signaling pathway in IL-1*β*-induced rat NP cells, which was also verified *in vivo* in a rat IDD model.

## 5. Conclusion

In the present study, we found that BBR enhanced cell survival of IL-1*β*-induced rat NP cells through promoting cell proliferation and inhibiting cell apoptosis and ECM degradation. BBR reversed IL-1*β*-induced damages in rat NP cells and alleviated IDD in a rat model by inducing autophagy through the AMPK/mTOR/Ulk1 signaling pathway. The present study might provide novel therapeutic potential against IDD.

## Figures and Tables

**Figure 1:** Berberine accelerates cell proliferation and suppressed apoptosis in IL-1*β*-induced NP cells. (a) NP cells were treated with 0, 0.13, 0.25, 0.50, 1.00, 2.00, 4.00, 8.00, and 16.00 *μ*M BBR for 7 days; then cell viability was detected by CCK-8 assay. (b) NP cells were treated with IL-1*β* in combination with 0, 0.25, 0.50, 1.00, 2.00, and 4.00 *μ*M of BBR; then cell viability was measured by CCK-8 on 0, 2, 4, and 6 days posttreatment. (c) NP cells were treated with 1.00 *μ*M BBR, IL-1*β*, or 1.00 *μ*M BBR combined with IL-1*β*, and cell viability was measured by CCK-8 on 0, 2, 4, and 6 days posttreatment. (d) NP cells were stained with BrdU and DAPI. (e) Relative BrdU-positive cells were counted and presented. (f) NP cells were treated with BBR alone or combined with IL-1*β*, and apoptosis were detected by FACS. (g) Percentage of apoptotic cells was presented. (h) NP cells were treated with BBR alone or combined with IL-1*β*, and protein expressions were analyzed by immunoblot. (i) Relative protein expression was analyzed by the ImageJ software. Scale bars: 25 *μ*m, magnified ×400. The data are shown as the mean ± SD of three experiments. ^∗^*P* < 0.05 compared with the IL-1*β* induced group; ^∗∗^*P* < 0.01 compared with the control group; ^##^*P* < 0.01 compared with the IL-1*β* induced group.

**Figure 2:** Effect of Berberine on ECM-related protein expression and ECM degradation in IL-1*β*-induced NP cells. (a) NP cells were treated with 1.00 *μ*M BBR, IL-1*β*, or 1.00 *μ*M BBR combined with IL-1*β*, and the mRNA level of aggrecan, collagen II, and MMP-13 was evaluated by RT-qPCR. (b) Confocal imaging of NP cells was collected by staining collagen II antibody (green). (c) Protein levels of aggrecan, collagen II, and MMP-13 were evaluated by immunoblot. Scale bars: 25 *μ*m, magnified ×400. The data are shown as the mean ± SD of three experiments. ^∗∗^*P* < 0.01 compared with control group; ^##^*P* < 0.01 compared with the IL-1*β* induced group.

**Figure 3:** Berberine activates autophagy in NP cells. (a, b) NP cells were treated with BBR, BBR and IL-1*β*, or BBR, IL-1*β*, and 3-MA (10 mM), (a) and protein expressions were analyzed by immunoblot. (b) Relative protein expression was analyzed by ImageJ software. (c) Confocal imaging of NP cells were collected by staining LC3II antibody (green). Scale bars: 25 *μ*m, magnified ×400. The data are present as the mean ± SD of three experiments. ^∗∗^*P* < 0.01 compared with the control group; ^##^*P* < 0.01 compared with the IL-1*β* group; ^&&^*P* < 0.01 compared with the BBR + IL-1*β* group.

**Figure 4:** Berberine induces autophagy by activating the AMPK/mTOR/Ulk1 signaling pathway in nucleus pulposus cells. (a, b) NP cells were treated with IL-1*β*, BBR and IL-1*β*, or BBR, IL-1*β*, and compound c (CC, AMPK inhibitor). (a) Protein expressions were measured by immunoblot and (b) the relative protein expression was analyzed by the ImageJ software. ^∗∗^*P* < 0.01 compared with the control group; ^##^*P* < 0.01 compared with the IL-1*β* group; ^&&^*P* < 0.01 compared with the BBR + IL-1*β* group.

**Figure 5:** Berberine ameliorates intervertebral disc degeneration *in vivo.* (a–c) Representative HE staining, Safranin O staining, and TUNEL staining of disc samples from different groups (arrows, TUNEL-positive) (scale bars: 25 *μ*m, magnified ×100). (b) The histological score and (c) relative ratio of TUNEL-positive cells are presented. (d, e) Protein expressions were measured by immunoblot and relative protein expression was analyzed by the ImageJ software. ^∗∗^*P* < 0.01 compared with the sham group; ^##^*P* < 0.01 compared with the IDD group.

## Data Availability

All data, models, and code generated or used during the study appear in the submitted article.

## Additional Points

*Highlights*. [1] BBR prevented IDD. [2] AMPK/mTOR/Ulk1 was a potential therapeutic target in IDD.
